# Activation of PERK-Nrf2 oncogenic signaling promotes Mdm2-mediated Rb degradation in persistently infected HCV culture

**DOI:** 10.1038/s41598-017-10087-6

**Published:** 2017-08-23

**Authors:** Yucel Aydin, Milad Chedid, Srinivas Chava, Donkita Danielle Williams, Shuanghu Liu, Curt H. Hagedorn, Suchitra Sumitran-Holgersson, Krzysztof Reiss, Krzysztof Moroz, Hua Lu, Luis A. Balart, Srikanta Dash

**Affiliations:** 1 Department of Pathology and Laboratory Medicine, New Orleans, Louisiana USA; 2 Department of Medicine, Division of Gastroenterology and Hepatology, New Orleans, Louisiana USA; 3 Department of Biochemistry, Tulane University Health Sciences Center, New Orleans, Louisiana USA; 4 Department of Medicinal Chemistry, College of Pharmacy, University of Utah, Salt Lake City, UT USA; 5 Department of Medicine and Genetics, University of Arkansas for Medical Sciences, Little Rock, Arkansas USA; 6 Laboratory of Transplantation Surgery and Regenerative Medicine, University of Gothenburg, Gothenburg, Sweden; 7 School of Medicine, LSU Health Sciences Center, New Orleans, Louisiana USA

## Abstract

The mechanism of how chronic hepatitis C virus (HCV) infection leads to such a high rate of hepatocellular carcinoma (HCC) is unknown. We found that the PERK axis of endoplasmic reticulum (ER) stress elicited prominent nuclear translocation of Nrf2 in 100% of HCV infected hepatocytes. The sustained nuclear translocation of Nrf2 in chronically infected culture induces Mdm2-mediated retinoblastoma protein (Rb) degradation. Silencing PERK and Nrf2 restored Mdm2-mediated Rb degradation, suggesting that sustained activation of PERK/Nrf2 axis creates oncogenic stress in chronically infected HCV culture model. The activation of Nrf2 and its nuclear translocation were prevented by ER-stress and PERK inhibitors, suggesting that PERK axis is involved in the sustained activation of Nrf2 signaling during chronic HCV infection. Furthermore, we show that HCV clearance induced by interferon-α based antiviral normalized the ER-stress response and prevented nuclear translocation of Nrf2, whereas HCV clearance by DAAs combination does neither. In conclusion, we report here a novel mechanism for how sustained activation of PERK axis of ER-stress during chronic HCV infection activates oncogenic Nrf2 signaling that promotes hepatocyte survival and oncogenesis by inducing Mdm2-mediated Rb degradation.

## Introduction

Approximately 3% of the world population is infected with hepatitis C virus (HCV)^1^. The majority of people infected with HCV develop chronic liver disease that often progresses to liver cirrhosis and hepatocellular carcinoma (HCC)^2–6^. Patients with cirrhosis have an increased risk to develop HCC^3, 4^. The highly effective DAA based antiviral therapy results in a high cure rate of chronic HCV infection^7, 8^. Additional versions of highly effective DAA combination therapies are expected to be available in the future, which provides hope that HCV infection can be globally eliminated^8^. This will require that all infected patients receive early diagnosis and access to antiviral treatment. However, chronically infected individuals who do not receive appropriate care have the highest risk of developing liver cirrhosis and HCC^9^. Some recently reported clinical studies show that HCV cure using DAA based antiviral therapy decreases HCC risk significantly among patients with advanced liver cirrhosis but does not eliminate the risk completely^10–12^. The risk of HCC persists for several years after viral cure among patients with advanced liver disease^9^. The mechanism of how chronic HCV infection causes hepatocellular carcinoma is unknown^13, 14^.

HCV is a positive-stranded RNA virus belonging to the *flaviviridae* family. The HCV genome is a single-stranded RNA molecule of 9600nts in length. The viral genome is translated in the endoplasmic reticulum into a large polyprotein, which is post-translationally processed by cellular and viral proteases into structural (core, E1 and E2) and non-structural proteins (NS2, NS3, NS4A, NS4B, NS5A and NS5B)^15, 16^. The viral mRNA translation and replication processes occur within the endoplasmic reticulum (ER), a membrane-enclosed organelle specific to eukaryotic cells. Sustained RNA translation and replication in the hepatocytes results in an accumulation of large amounts of viral proteins in the ER, which generates a substantial amount of stress response called ER-stress^17, 18^. The low level accumulation of misfolded or unassembled proteins in the ER is cleared by ubiquitination and proteosomal degradation pathway called ER-associated degradation (type I). When this mode of protein degradation is not sufficient, the ER initiates a second line of protein degradation mechanism through induction of UPR-mediated autophagy (type II). Chronic ER-stress activates several well-orchestrated cellular transcription programs, called unfolded protein response (UPR), in order to restore cellular homeostasis and prevent cell death^19^. The UPR is orchestrated by three different cellular transcription factors: protein kinase-like endoplasmic reticulum kinase (PERK), activation of transcription factor 6 (ATF6), and inositol requiring enzyme 1 (IRE1), to maintain ER homeostasis^18^. Long-term ER-stress induces macroautophagy, and the UPR can regulate expression of autophagy genes and autophagosome formation. We and many other researchers have shown that acute HCV infection induces UPR and autophagy response to promote cell survival^20–35^. To understand the significance of ER-stress in chronic liver disease and liver cirrhosis, the expression levels of UPR genes were examined using liver biopsies from chronically infected patients plus explant cirrhotic livers with HCC^33–35^. These findings show that ER-stress persists during chronic liver disease, liver cirrhosis and HCC, suggesting that chronic ER-stress plays a major role in HCC development.

The detailed mechanism of how chronic ER-stress induces liver injury and HCC is not fully understood. The hepatic UPR activation during HCV infection is associated with the increased production of reactive oxygen intermediates (ROI) from the mitochondria due to calcium release from the ER^22^. A number of studies have shown that HCV infection induces oxidative stress through Ca^++^signaling in the ER^23–25^. Several HCV proteins including core, E1, E2, NS3, NS4A and NS5A induce oxidative stress and induce cytoprotective genes harboring a short cis-acting sequence, the antioxidant response elements (ARE) in their promoters^36^. The antioxidant response is mainly mediated by NF-E2 related factor 2 (Nrf2) activation and binding to the ARE elements in the nucleus. The activation of Nrf2 through phosphorylation is mediated by a number of kinases including protein kinase C (PKC), phosphoinositide-3-kinase (PI3K), mitogen activated kinase (p38 and ERK1/2) and casein kinase 2 (CK2)^37–41^. The activation of cytoprotective Nrf2 signaling during HCV infection generated conflicting reports since most of these studies have been done in a short-term acute HCV infection model. The exact role of UPR/oxidative stress and Nrf2 activation during chronic HCV infection is unclear.

We performed this study to understand how chronic ER-stress contributes to oncogenic Nrf2 signaling in a persistently infected cell culture system in primary human hepatocytes and Huh-7.5 cells. In this study, we show that chronic ER-stress/UPR response during persistent HCV infection resulted in activation of Nrf2 and its nuclear translocation being mediated by PERK axis of the UPR. Our results suggest that persistent HCV infection induces Nrf2/ARE dependent expression of oncoprotein Mdm2 for cell survival. We report here that HCV induced ER-stress response promotes Mdm2-mediated proteosomal degradation of retinoblastoma protein (Rb). Our results provide a potential mechanism by which oncogenic Nrf2 signaling contributes to HCC development during chronic HCV infection.

## Materials and Methods

### Primary human hepatocytes (PHHs)

PHHs were obtained from XenoTech LLC, Kansas City, MO, and cultured with hepatocyte culture media supplemented with 10% human serum (Invitrogen, Brown Deer, WI). After 24 hours they were infected with cell culture grown HCV-GFP chimera virus with a MOI (multiplicity of infection) of 0.1 described earlier^42^. After 18 hours of infection, hepatocytes were replaced with fresh hepatocyte culture media (XenoTech, LLC, Kansas City, MO) supplemented with 10% human serum (Invitrogen, Brown Deer, WI). Uninfected or infected PHHs were harvested every 3 days and cell pellets were used for RNA isolation and Western blot analysis. The success of HCV replication in the infected PHHs was assessed by the detection of positive strand HCV RNA levels by reverse transcription real-time quantitative PCR (QRT-PCR) and Western blot analysis of HCV NS3 protein.

### Cell Culture and Chemicals

Huh-7.5 cells were obtained from Charles M. Rice (Rockefeller University, New York). The Huh-7.5 cell line was maintained in Dulbecco’s Modified Eagle’s Medium (DMEM) supplemented with 2 mM L-glutamine, sodium pyruvate, nonessential amino acids, 100 U/mL penicillin, 100 μg/mL streptomycin, and 10% fetal bovine serum. Huh-7.5 cells were infected with JFH1-GFP chimera HCV using a protocol developed in our laboratory as previously described^31^. Recombinant human IFN-α was purchased from Schering Plough, Kenilworth, NJ. Sofosbuvir was obtained from Acme Biosciences, Inc. (Palo Alto, CA) and ledipasvir was obtained from Selleck Chemicals (Houston, TX). Thapsigargin (TG), tauroursodeoxycholic acid (TUDCA), PERK inhibitor (GSK 2606414), α-tocopherol, and roscovitine were obtained from Sigma-Aldrich (St. Louis, CA). Antibody to pNrf2 was purchased from Abcam. Antibodies to GRP78 (BiP), PERK, eIF2α, peIF2α, CHOP, IRE1, GFP and Rb were obtained from Cell Signaling (Beverly, MA). Antibody to NS3 was purchased from Virogen Inc. Antibodies to HCV core and pIRE1 were purchased from Thermo Scientific. Antibody to GRP94, GADD34, pPERK, ATF4, XBP1, ATF6, Mdm2, β-actin and GAPDH were purchased from Santa Cruz Biotechnology (Santa Cruz, CA).

### SDS-PAGE and Western blotting

Infected Huh-7.5 cells were harvested by the treatment of trypsin-EDTA. Cells were lysed in ice-cold lysis buffer (50 mM Tris HCl pH 8.0, 140 mM NaCl, 1.5 mM MgCl2, 0.5% NP-40 with complete protease inhibitor from Invitrogen) for 10 minutes in ice (about 1 × 10^6^ cells/200μL). Whole cells and cell debris were pelleted by low-speed centrifugation and cleared supernatants were transferred to a new tube. Protein concentration was determined by DCA protein assay. Samples were boiled for 10 minutes at 80 °C in the presence of 1X SDS-PAGE-loading buffer (250 mM Tris-HCL pH 6.8, 40% glycerol, 8% SDS, 0.57M β-mercaptoethanol, 0.12% bromophenol blue). Approximately 20 μg of protein was loaded onto 12% SDS-PAGE and transferred into a nitrocellulose membrane (Thermo Scientific). The membrane was blocked using solution containing 5% of blotting-grade milk power (Bio-Rad, Hercules, CA) for 2 hours then incubated with a primary antibody. After overnight incubation, the antigen-antibody complex was visualized with HRP-conjugated goat anti-rabbit or anti-mouse IgG and the ECL detection system (Amersham).

### Detection of Reactive Oxygen Species (ROS)

Production of ROS was measured by using the cell-permeant H2DCFDA (Thermo Fisher) according to the manufacturer’s instructions. The 2′, 7′-dichlorodihydrofluorescein diacetate (H2DCFDA) fluorescent probe reacts with ROS including hydrogen peroxide and hydroxyl radicals. The cell-permeant H2DCFDA diffuses into cells and is retained in the cytoplasm after cleavage by intracellular esterases. The ROS converts the nonfluorescent H2DCFDA to the highly fluorescent 2′, 7′-dichlorofluorescein (DCF), which can be detected by a fluorescent microscopy or quantified by flow cytometry. The oxidation-reduction potential of HCV infected culture supernatants at day 12 was compared with uninfected cell supernatants using a novel galvanostat-based technology (MiOXSYS^TM^ System; Aytu Bioscience, Englewood, CO, USA). Briefly, 30 µl of supernatants was exposed to the MiOXSYS sensor. The MiOXSYS system provides an estimation of the static oxidation-reduction potential (sORP), measured in mV. It represents the integrated measure of the existing balance between total oxidants and reductants in a biological system.

### Flow Cytometry Analysis

The number of GFP expressing cells in the HCV infected Huh-7.5 cells were determined by flow cytometry using a BD FACSCalibur machine (BD Bioscience). The number of cells progressing through S-phase was determined by flow analysis after PI staining (BD-Biosciences).

### Immunohistochemical staining

Tissue culture cells were immobilized onto a glass slide via the cytospin centrifugation method. Immunostaining of the cytospin slides was performed using a standard protocol established in our laboratory^35^. Immunostaining of paraffin embedded tissue sections was carried out using a standard method established in the laboratory^34^.

### SiRNA transfection

Persistently HCV infected Huh-7.5 cells were cultured in 6-well plates (up to 60% confluence in DMEM supplemented with 10% FBS media) without antibiotics. The next day, culture media was replaced with fresh DMEM with 2% FBS and cells were then transfected with siRNA to either Mdm2 (siRNA1: 5′-GCCUGGCUCUGUGUGUAAU-3′, siRNA2: 5′-GCCCUGCCCAGUAUGUAGA-3′)^43^ Nrf2 (siRNA1: 5′-GAAUGGUCCUAAAACACCA-3′, siRNA2: 5′-UGACAGAAGUU GACAAUUA-3′)^44, 45^ or PERK (5′-CAAGAGGAAGACAUCCUGCTT-3′)^46^ or ATF6 (5′-GCAACCAAUUAUCAGUUUATT-3′)^47^ or IRE1 (5′-GGACGUGAGCGA CAGAAUATT-3′)^48^ using Lipofectamine (Life Technology, Grand Island, NY). Knockdown efficiency was analyzed by Western blot analysis.

### Statistical analysis

The immunostaining and immunofluorescence images were quantified using a computer image analysis software package (ImageJ NIH, Bethesda, MD)^49, 50^. All measurements were made at least in triplicate (n = 3). To compare means within groups we performed one factor analysis of variance (ANOVA) using the GraphPad Prism software. We assumed that all measurements have normal probability distributions, which is expected for these types of data. When the overall p-value for the ANOVA analysis was significant (p < 0.05), we applied Dunnet’s post hoc test to compare control samples with experimental samples. When performing comparisons between multiple groups, each analyzed with ANOVA, we used the Bonferroni correction to determine a revised cutoff for statistical significance that gives a combined 5% type I error probability. *P < 0.05, **P < 0.001, ***P < 0.0001.

## Results

### Persistent HCV replication induced chronic ER-stress

HCV is a RNA virus that develops high rate of chronic infection in hepatocytes. In this study, we examined the long-term impact of HCV replication on ER-stress and cell survival using non-proliferative primary human hepatocytes (PHHs). PHHs seeded in a six well tissue culture plate were infected with HCV-NS5A-EGFP reporter virus (MOI 0.1) (JFH1-AM120) overnight. Replication of HCV in PHHs model was confirmed by the measurement of viral NS3 protein, NS5A-green fluorescence (GFP) fusion protein by Western blot analysis over 18 days **(**Fig. 1A **)**. The highly permissive Huh-7.5 cells based infection model was also used as an alternative method to investigate the impact of high-level persistent HCV replication of cellular ER-stress response and cell survival. Huh-7.5 cells were infected with JFH-AM120 (MOI 0.1) and HCV replication was studied over 21 days by the measurement of HCV NS3 and GFP expression. Western blot analysis found an increased expression of HCV NS3 protein in infected Huh-7.5 cells over 21 days **(**Fig. 1B **)**. These results are supported by expression of NS5A-GFP fusion protein by fluorescence microscopy with nuclear DAPI staining. We show that Huh-7.5 cells infected with JFH-AM120 show increased expression of NS5A-GFP **(**Fig. 1C **)**. Quantifications of GFP positive cells by ImageJ software show that the level of HCV replication was increased with time **(**Fig. 1D **)**. After HCV infection, the percentage of Huh-7.5 cells expressing GFP was analyzed by flow cytometry analysis at 0, 9 and 12 days. These results indicate HCV infection was 42% at day 9, which was increased in time with more than 97% of cells were GFP positive at day 12. These results confirmed the high-level replication of JFH-AM120 chimera virus in non-transformed (PHHs) and transformed Huh-7.5 cells.

**Figure 1:** Shows level of HCV replication in non-proliferative primary human hepatocytes and proliferative Huh-7.5 cell cultures. PHHs were infected with HCV-GFP virus (JFH-AM120) at a MOI of 0.1 by overnight incubation. The next day cells were incubated with fresh media with 10% human serum. **(A)** HCV replication in PHHs model was confirmed by the measurement of NS3 and NS5A-GFP fusion protein levels by Western blot. **(B)** Western blot analysis showed time dependent increase in the expression of NS3 protein in Huh-7.5 cells infected with HCV-GFP virus. **(C)** Expression of NS5A-GFP chimera protein with DAPI staining in Huh-7.5 cells infected with HCV-GFP virus over 12 days. **(D)** Quantification of NS5A-GFP expression by ImageJ software. **(E)** Flow cytometry analysis shows expression of GFP in infected Huh-7.5 cells at day 0, 9 and 12 days. Fluorescence images shown in panel C were taken at 40X magnification.

HCV is a positive-stranded RNA virus in which viral translation, replication and assembly occur mostly at the rough ER and ER derived membranes. Accumulation of large amounts of viral proteins during persistent replication induces stress response in infected cells. Most of the prior studies have shown that the UPR was either partially activated or suppressed to attenuate the ER-stress-mediated hepatocellular apoptosis using transformed hepatoma cell culture system (Huh-7.5) cells soon after virus infection^21–27^. It is unclear whether persistent HCV replication induced chronic or adaptive ER-stress in untransformed hepatocytes. The unfolded response (UPR), a cellular transcriptional program, starts due to ER-stress with the activation of eukaryotic translation initiation factor 2a kinase 3 (PKR-like ER kinase; PERK), serine/threonine-protein kinase/endonuclease (IRE1) and cyclic AMP-dependent transcription factor (ATF6) following removal of the chaperone binding immunoglobulin protein (BiP) **(**Fig. 2A **)**. Using HCV infected PHHs model, we found that the expression of all three branches of UPR are induced and autophagy markers were also induced by Western blot analysis for 18 days **(**Fig. 2B **)**. We noticed that the expression of UPR markers remained high in the infected culture over 18 days as compared to uninfected PHHs, indicating that HCV replication induces chronic ER-stress. We did not see any significant activation of ER-stress markers in uninfected PHHs when cultured for similar time points without HCV infection (data not shown). The status of ER-stress/UPR response was examined by comparing the expression of BiP, PERK, ATF6α and IRE1α in Huh-7.5 cells after HCV infection for over 21 days **(**Fig. 2C **)**. We noticed that the activation of pNrf2 is stronger and faster in infected PHHs because these cells do not express p62. Whereas Huh-7.5, a cancer cell line, expresses p62, therefore basal level of Nrf2 activation is seen prior to infection. During early state, up to day 6 after HCV infection, p62 is degraded because of autophagy induction. Due to this reason, we see a delay in Nrf2 activation and nuclear accumulation starting at day 9, when cells are negative for p62. These results are consistent with PHHs, which indicate that HCV infection induces chronic ER-stress and UPR response.

**Figure 2:** HCV infection activates ER-stress response and induces expression of numerous UPR genes for cell survival in infected PHHs and Huh-7.5 cells. **(A)** Illustrates the mechanisms for how HCV protein accumulation induces ER-stress and activates three branches of UPR gene expression. **(B)** Cell lysates prepared from infected PHHs were examined for the expression of ER-stress chaperone, Nrf2 activation; UPR genes (PERK, ATF6 and IRE1) by Western blot analysis. **(C)** UPR gene expression and Nrf2 activation in Huh-7.5 cells after HCV infection.

### Persistent HCV infection activates Nrf2 activation through ER-stress/PERK signaling

A number of investigators have shown that HCV infection also induces oxidative stress and accumulation of reactive oxygen species through calcium release from the ER^22–25^. Intracellular ROS levels between uninfected and persistently HCV infected culture was monitored using a fluorescent-based detection method **(**Fig. 3A **)**. In this assay, H2DCFDA is converted to the highly fluorescent 2’7’-dichlorofluorescein due to the presence of ROS. The fluorescence intensity is proportional to the amount of oxidant present in HCV infected cells. The oxidative stress was significantly high in HCV infected culture as compared to uninfected Huh-7.5 cells **(**Fig. 3B **)**. A flow cytometric analysis based quantitative approach shows that the majority of cells infected with HCV show punctate fluorescence staining, due to presence of high oxidative stress response **(**Fig. 3C **)**. Cellular H2O2 levels were also determined using OxiSelect hydrogen peroxide/peroxide assay **(**Fig. 3D **)**. An essential factor involved in the defense against oxidative stress is the NF-E2 related factor 2 (Nrf2) that is activated in response to oxidative stress. It induces varieties of cytoprotective genes harboring a short cis-acting sequence called the antioxidant response element (ARE) in their promoter^51^. The transcription factor Nrf2 plays an essential role in the control of ARE-regulated genes. We examined the nuclear translocation of Nrf2 in persistently infected culture in a kinetic study by immunocytochemical staining **(**Fig. 4A **)**. We found predominant nuclear accumulation of Nrf2 in 100% of HCV infected culture starting from day 9, suggesting that HCV replication promotes nuclear translocation. The expression of HCV core correlated well with the Nrf2 nuclear translocation **(**Fig. 4B **)**. An ARE-based reporter assay was performed to measure the impact of HCV replication on the activation of luciferase expression^38^. Persistently infected Huh-7.5 cells at day 12 were transfected with ARE-Renilla Luciferase, and the activation of ARE-promoter in the presence and absence of HCV replication was measured. The reporter assay shows that persistent HCV infection significantly activates ARE-mediated luciferase expression **(**Fig. 4C **)**. These results support the notion that Nrf2 antioxidant property is predominantly mediated by nuclear translocation and ARE-mediated gene transcription.

**Figure 3:** Oxidative stress response in persistently HCV infected Huh-7.5 cells. **(A)** Oxidative stress due to generation of ROS was measured using conventional fluorescence microscopy. In this assay, the nonfluorescent dye (H2DCFDA) is oxidized to a fluorescence green (DFA) by ROS only in HCV infected cells. Uninfected cells show no fluorescence. **(B)** Quantification of fluorescent intensity in three different areas of uninfected and infected culture was measured by ImageJ software. Fluorescence values are proportional to intracellular ROS. **(C)** Flow cytometric analysis of oxidized fluorescence of uninfected and infected Huh-7.5 cells. **(D)** Relative Oxidation-Reduction Potential (ORP) of cell free media of uninfected and HCV infected Huh-7.5 cells.

**Figure 4:** Persistent HCV replication induces Nrf2 activation and nuclear translocation. **(A)** Immunocytochemical staining of HCV core and pNrf2 in HCV infected Huh-7.5 cells at different days after HCV infection. **(B)** Quantification of core positive and Nrf2 positive infected Huh-7.5 cells, three high-power fields were measured using ImageJ software. ***P < 0. 0001. **(C)** Activation of ARE-luciferase reporter in uninfected and HCV infected cells at day 12. Two different concentrations of ARE-luciferase plasmid were transfected to Huh-7.5 cells and infected Huh-7.5 cells. After 24 hours, equal amounts of protein lysates were measured for luciferase activity. The luciferase values were normalized to one microgram of protein.

### Nuclear translocation of Nrf2 promotes Mdm2-mediated Rb degradation

We examined whether Nrf2 nuclear translocation confers cytoprotection against oxidative stress by tumor suppressor degradation. Diverse signaling pathways have been established in mammalian cells to regulate expression of tumor suppressor Rb and p53 to improve cell survival pathway^52–54^. Mdm2 is an E3 ubiquitin ligase that promotes p53 ubiquitination at several lysine residues, leading to its proteosomal degradation^54^. In many cancer models, Mdm2 expression is regulated by a negative feedback loop for maintaining low p53 levels^54^. We showed that chaperone-mediated autophagy (CMA) is induced during persistent HCV infection and degrades p53 in a lysosomal dependent manner by binding to Hsc70^35^. CMA is induced as a cell survival mechanism in response to oxidative stress in Nrf2 dependent mechanism^55–57^. A recent study showed the presence of putative ARE elements located in the first intron is responsible for Mdm2 promoter activity^58^. In this study, we examined whether the Nrf2-mediated induction of Mdm2 expression could promote Rb degradation. Confocal image analysis of persistently infected Huh-7.5 cells was performed to confirm that HCV expression induces Mdm2 expression and degrades Rb expression **(**Fig. 5A **)**. Image analysis-based quantification shows that HCV infection significantly induced Mdm2 expression and Rb levels were reduced in HCV replicating cells **(**Fig. 5B **)**. To clarify this novel mechanism, Western blot analysis was performed to examine the expression levels of Mdm2 and Rb in HCV infected PHHs and persistently HCV infected Huh-7.5 cells **(**Fig. 5C and E **)**. To determine the statistical correlation coefficient between Mdm2 and Rb expression, fraction of variance denoted by R^2^ values was determined (Fig. 5D and F). In our analysis, the R^2^ values are very close to 1.0 suggesting that the induction of Mdm2 perfectly predict the degradation of Rb in HCV infected PHHs and Huh-7.5 cells. Real-time RT-PCR data showed that HCV infection did not alter Rb mRNA levels in Huh-7.5 cells. Persistent HCV infection induced mRNA expression of Mdm2 in both PHHs and Huh-7.5 cells **(**Fig. 5G and H **)**. A strong inverse correlation between the expression of Mdm2 and Rb proteins was observed in infected PHHs and Huh-7.5 cells, suggesting that Mdm2 regulates the expression of Rb during persistent HCV infection.

**Figure 5:** Persistent HCV replication induces Mdm2-mediated degradation of Rb tumor suppressor. **(A)** Colocalization studies by confocal microscopy between HCV-GFP and nuclear expression of Mdm2 and Rb in infected Huh-7.5 cells at day 12. **(B)** Fluorescence intensity of three areas was measured by ImageJ software, indicating HCV infection induces Mdm2 but degrades Rb. **(C)** Cell lysates were prepared from infected PHHs at indicated time points, and were examined for the expression of Mdm2 and Rb by Western blotting. GAPDH levels were examined for comparison. **(D)** Band intensities of Mdm2 and Rb were measured using ImageJ software andR^2^ values were determined by excel software. (**E**) The expressions of Rb and Mdm2 were measured in the infected Huh-7.5 cells at indicated time points by Western blotting. (**F**) Band intensities of Mdm2 and Rb were measured using ImageJ software and R^2^ values were determined by excel software. **(G)** Real-time RT-PCR analysis of Rb mRNA levels of HCV infected Huh-7.5 cells. Rb forward sequence 5′-GGAAGCAACCCTCCTAAACC-3′, reverse sequence 5′-TTTCTGCTTTTGCATTCGTG -3′. (**H**) Real-time RT-PCR shows that Mdm2 mRNA levels are induced in HCV infected PHHs and Huh-7.5 cells. Mdm2 forward sequence 5′-TGTAAGTGAACATTCAGGTG-3, reverse sequence 5′-TTCCAATAGTCAGCTAAGGA-3′. ***P value < 0.0001.

### Mdm2-mediated Rb degradation induces genomic instability and aneuploidy in persistently infected culture

Genomic instability is a common characteristic of many cancers, which most often occurs in the absence of p53 and Rb tumor suppressor^59, 60^. It has been reported that 30–60% of human hepatocellular carcinoma show inactivation of Rb and p53 tumor suppressors^60^. Previous studies have shown that Mdm2 overexpression leads to increased chromosome/chromatid breaks, centrosome hyper amplification and aneuploidy^61, 62^. We reported that HCV-induced stress response degrades wild type and mutant p53 by chaperone-mediated autophagy^35^. Our results show that HCV-induced stress response also degrades Rb tumor suppressor through Mdm2-mediated proteosomal degradation. The tumor suppressor Rb has important roles in variety of biological processes including cell cycle, DNA synthesis, DNA damage, DNA repair, senescence, apoptosis and cancer development^63^. A key function of Rb is to bind to E2F proteins, forming active transcription repressor complexes that block expression of genes involved in DNA replication and cell cycle progression^64^. To understand the impact of Mdm2 over expression for cellular growth, both uninfected and HCV infected cells were grown in normal growth media for six days and cell numbers were counted daily. Results were expressed as the mean of three independent experiments **(**Fig. 6A **)**. One of the initiating events of oncogenesis is tetraploidization, that is generation of cells that contain twice as much DNA and chromosomes than their normal diploid counterparts. In addition, tetraploid cells can undergo a subsequent depolyploidization cascade that results in rampant aneuploidy due to multipolar division. Cells that illicitly survive these checkpoints are prone to chromosomal instability and aneuploidization^65^. Diploid, tetraploid and aneuploid populations were analyzed between uninfected and HCV infected cells to understand the impact of Mdm2-mediated Rb degradation on cell cycle. We found increased existence of tetraploidy populations in persistently HCV infected cells due to increased Mdm2 expression and loss of Rb **(**Fig. 6B **)**. HCV-induced Mdm2-mediated Rb degradation resulted in an increased fraction of infected cells in S phase of cell cycle **(**Fig. 6C **)**. Silencing Nrf2 in the HCV infected culture reversed the S-phase cell cycle entry from 71.6% to 44.7% and decreased tetraploidy population. These results suggest that ER-stress associated with persistent HCV infection stimulates cell cycle progression through Mdm2-mediated Rb degradation.

**Figure 6:** Persistent HCV replication in Huh-7.5 cells promotes cell growth and S-phase entry **(A)** HCV infected Huh-7.5 cells and uninfected cells were grown in normal growth media for 6 days. Cell numbers were counted daily. Results were shown as mean and standard error from three different experiments. **(B)** Show percentage of S-phase cells in diploid and tetraploid cell population. Rb loss in HCV culture shows an increase in tetraploidy population. Nrf2 silencing using two siRNAs in infected culture decreased tetraploidy population. **(C)** HCV infected (day 12) and uninfected Huh-7.5 cells were subjected to cell cycle analysis after propidium iodide staining. There is an increase in S-phase of cell cycle due to Rb loss in HCV infected cells. Silencing Nrf2 using two siRNAs decreased S-phase population.

### ER-stress inducer promotes Mdm2-mediated Rb degradation

The Mdm2-mediated regulation of Rb degradation was confirmed in the presence of ER-stress inducer (TG) and ER-stress inhibitor (TUDCA). Persistently infected Huh-7.5 cells and one immortalized, non-transformed fetal liver derived cell line were treated with increasingly viable concentrations of TG for 24 hours, then expression of Mdm2 and Rb level were examined by Western blot analysis **(**Fig. 7A and B). The expression level of Mdm2 and Rb protein was examined in the same cell line in the presence of ER-stress inhibitor. TUDCA, by Western blot analysis **(**Fig. 7C and D). Previously, we showed that silencing Mdm2 expression in HCV infected culture did not restore p53 levels^35^. In this study, we found that silencing Mdm2 expression by siRNA in persistently infected Huh-7.5 cells (day 15) restored Rb expression **(**Fig. 7E **)**. Inhibition of Mdm2 expression by roscovitine restored Rb degradation in HCV infected Huh-7.5 cells **(**Fig. 7F **)**. Mdm2-mediated degradation of Rb in HCV infected culture is inhibited by proteasome inhibitor MG132, suggesting that proteasome-dependent Rb degradation promoted by Mdm2 **(**Fig. 7G **)**.

**Figure 7:** Western blot analysis shows the effect of ER-stress inducer (TG), inhibitor (TUDCA) and siRNA mediated silencing of Mdm2 on the expression of Rb in HCV infected and uninfected hepatic cells. **(A)** HCV infected Huh-7.5 cells were treated with variable concentrations of TG. After 24 hours, the expression of Mdm2 and Rb expression were examined by Western blot analysis. **(B)** Similar analysis was performed using an immortalized human hepatocyte cell line (HTERT) after treatment with TG. **(C)** HCV infected cells were treated with ER-stress inhibitor (TUDCA). The expression of Mdm2 and Rb levels were examined by Western blot. The expressions of PERK and Nrf2 were measured using the same lysate **(D)** TUDCA treatment of uninfected immortalized human hepatocytes **(E)** Silencing Mdm2 restores Rb expression. **(F)** Cyclin dependent kinase (CDK) inhibitor, roscovitine inhibits Mdm2 and restores Rb expression in HCV infected culture. **(G)** Pre-treatment with proteasome inhibitor (Mg132) restores Mdm2-mediated Rb degradation.

### Silencing PERK and Nrf2 pathways restore Mdm2-mediated Rb degradation

Persistent HCV replication induces sustained nuclear translocation of Nrf2 and activation of ER-stress and oxidative stress response. We used siRNA based silencing experiments to determine, which branch of ER-stress is responsible for Mdm2-mediated Rb degradation. At day 15, infected Huh-7.5 cells were treated with different siRNAs targeted to PERK, ATF6 and IRE1 branch of UPR. After 72 hours, cell lysates were examined for Mdm2 and Rb protein expression by Western blot analysis. Silencing IRE1 and ATF6 did not reduce the expression of Mdm2 and did not restore Rb expression levels **(**Fig. 8A and B **)**. Silencing PERK pathway showed decreased expression of Mdm2 and induced Rb expression, suggesting that persistent HCV infection induces Mdm2-mediated Rb degradation using PERK branch of UPR **(**Fig. 8C **)**. Persistently HCV infected Huh-7.5 culture treated with PERK inhibitor showed decreased expression of Mdm2 and increased expression of Rb **(**Fig. 8D **)**. PERK silencing also showed reduced activation of Nrf2. Silencing PERK had no effect of HCV core protein expression **(**Fig. 8E **)**. All these data are consistent with the activation of Nrf2 in persistently infected culture measured by Western blot analysis (Fig. 2B and C **)**. The expression of PERK, ATF6, IRE1, Mdm2, Nrf2 levels were comparable between infected culture that were transfected with scramble siRNA or siRNA targeted to GAPDH (Fig. 8F). Taken together these results suggested that HCV induced PERK activation promotes nuclear translocation of Nrf2, leading to increased expression of Mdm2 and decreased expression of Rb. The Nrf2 mediated Mdm2 gene expression is required to improve cell survival pathways to overcome the stress response associated with persistent HCV replication.

**Figure 8:** Activation of Mdm2/Rb degradation by ER-stress. HCV infected cells were treated with different concentrations of siRNAs targeted to three branches of UPR using lipofectamine. After 72 hours, cell lysates were prepared and 20 µg of proteins were loaded on to SDS-PAGE. The expressions of Mdm2 and Rb levels were examined by Western blotting. **(A)** Knockdown efficiency of IRE1α and its impact on the expression levels of Mdm2/Rb. **(B)** Knockdown efficiency of ATF6α and its impact on the expression levels of Mdm2/Rb. **(C)** Knockdown efficiency of PERK and its impact on the expression levels of Mdm2/Rb. The expressions of Nrf2 and pNrf2 were examined in the same lysate. **(D)** Western blot for Mdm2, Rb and Nrf2 activation of HCV infected cells treated with PERK inhibitor. (**E**) Knockdown efficiency of Nrf2 and its impact on the expression levels of Mdm2/Rb. The expression of HCV core did not change during the siRNA treatment. (**F**) The levels of PERK, IRE1, ATF6, Mdm2 and Nrf2 levels were not altered in the cells transfected with scrambled siRNA or GAPDH siRNA.

### PERK-dependent activation of Nrf2 signaling in persistent HCV infection

Current data shows that Nrf2 phosphorylation is mediated by a number of protein kinases including protein kinase C (PKC), phosphoinositide-3-kinase (PI3K), mitogen-activated protein kinases (p38 and ERK1/2), casein kinase 2 (CK2) and PERK pathway^36–41^. To determine which kinases block the nuclear translocation of Nrf2 in persistently infected culture, the ER-stress inhibitor TUDCA, PERK inhibitor and antioxidant (α-tocopherol) were added to HCV infected culture for 72 hours and then nuclear translocation was examined by immunostaining **(**Fig. 9A **)**. The signal was quantified by ImageJ software indicating that only ER-stress inhibitor and PERK inhibitor were able to prevent Nrf2 nuclear translocation **(**Fig. 9B **)**. Treatment with α-tocopherol (Vitamin E) did not prevent Nrf2 activation and nuclear translocation in HCV infected Huh-7.5 cells. These data demonstrate that persistent HCV infection promotes Nrf2 nuclear translocation and expression of genes involved in cell survival pathways in response to ER-stress through PERK pathway. We then compared whether HCV clearance induced by antiviral therapy could result in resolution of viral-induced Nrf2 activation and nuclear translocation in persistently infected culture. Infected cells at day 12 were given two rounds of antiviral treatment using either IFN-α or Sofosbuvir or Ledipasvir or combination of both (Harvoni). Then, nuclear translocation of Nrf2 was examined by immunostaining **(**Fig. 9C **)**. The intensity of Nrf2 staining in the nucleus was quantitatively measured by ImageJ software, which showed that only IFN-α based antiviral therapy is able to prevent activation of Nrf2 signaling and nuclear translocation **(**Fig. 9D **)**. These data are consistent with our previous observation indicating that DAAs themselves induce ER-stress, which is why the Nrf2 activation was not prevented after HCV clearance^35^. In order to evaluate the oncogenic effects of Nrf2 signaling on Mdm2 and Rb expression in HCV related HCC, immunohistochemical staining of Nrf2, was performed using five HCV infected cirrhotic liver with HCC. A prominent nuclear translocation of Nrf2 was seen in most of the tumor area as compared to non-tumorous cirrhotic liver **(**Fig. 10 **)**. These results suggest that Nrf2 activation and nuclear translocation plays an important role in HCC mechanism induced by chronic HCV infection.

**Figure 9:** The effect of ER-stress inhibitors and oxidative stress inhibitors on Nrf2 nuclear translocation and HCV replication. Persistently HCV infected Huh-7.5 cells were treated with ER-stress inhibitor TUDCA, PERK inhibitor, and an anti-oxidant (α-tocopherol) for 72 hours. After this treatment, cells were harvested by trypsin-EDTA, washed with PBS, and immobilized onto glass slide by cytospin method. Immunostaining for HCV core and pNrf2 was performed. **(A)** Shows the nuclear translocation of pNrf2 in HCV infected Huh-7.5 cells with different inhibitors. Short-term treatment with inhibitors did not change HCV core expression. **(B)** Shows the quantification core and Nrf2 nuclear translocation after different inhibitors by ImageJ software. **(C)** Impact of HCV clearance by DAA treatment on the Nrf2 nuclear translocation. HCV infected Huh-7.5 cells day 12 were given two rounds of antiviral treatment with IFN-α, sofosbuvir, ledipasvir or combination of sofosbuvir plus ledipasvir. After 72 hours, cells were split, and then treated again with the same antiviral agent. After two rounds of antiviral treatment, the expressions of HCV core and pNrf2 were measured by immunostaining. **(D)** Shows the quantification core and Nrf2 nuclear translocation after antiviral treatments by ImageJ software.

**Figure 10:** The expression of Nrf2 was examined using paraffin-embedded tissue sections of five HCV infected cirrhotic liver with HCC by immunohistochemical staining. Nuclear translocation of Nrf2 was seen only in the tumor areas of HCV infected liver cirrhosis with HCC. Most of the non-tumorous hepatocytes in the cirrhotic liver show negative nuclear Nrf2 staining.

## Discussion

Chronic HCV infection is the leading cause of liver cirrhosis and hepatocellular carcinoma (HCC) in the United States and many Western countries. Additional risk factors, such as hepatitis B virus or HIV coinfection, obesity, insulin resistance, alcoholic and non-alcoholic liver diseases trigger HCV-related HCC progression. Availability of a highly effective DAA-based antiviral strategy is expected to induce high rates of HCV clearance and decrease the incidence of HCC related to HCV infection. The risk of HCC development will not be completely eliminated in individuals with liver cirrhosis, so these patients need continuous surveillance for cancer risk. The mechanism showing how host-virus interaction results in development of liver cirrhosis and cancer is unknown. Understanding the HCV induced carcinogenic mechanisms may also increase our understanding of how non-viral etiologies promote HCC. Significant progress has been made regarding the genetic alterations and activation of oncogenic signaling that influence the survival of cancer cells by suppressing apoptosis and cell cycle regulation. Activation of oncogenes, oxidative stress/ER-stress and the role of tumor suppressor genes such as retinoblastoma, p53 gene, and Mdm2 pathway are involved in HCC development^66^.

Accumulating evidence suggests a close relationship between chronic HCV infection, oxidative stress, and liver disease progression. A review describes that HCV replication induces Ca^++^ release by ER-stress mechanisms, which leads to generation of reactive oxygen species (ROS) in infected cells, leading to oxidative stress^23^. Infected cells initiate a cytoprotective mechanism to protect cells against harmful effects of ER-stress induced cell death. Most of the cellular cytoprotective machinery stems from unfolded protein response generated due to ER-stress. One of the antioxidant transcription factors regulated by PERK axis of UPR is Nrf2, which protects liver cells from oxidative stress generated by persistent viral infection or non-viral insults^41^. Recent studies have found many other cellular kinases also phosphorylate Nrf2, leading to its activation and nuclear translocation^36–41^. The Nrf2 pathway has been implicated as a cytoprotective mechanism against not only oxidative stress but also cell survival and liver cancer development^67, 68^. At present, three different groups have published conflicting data on the activation of Nrf2 mediated cytoprotective response during HCV infection^36, 38, 69^. The first two reports, by Burdett *et al*.^38^ and Ivanov *et al*.^36^ claim that HCV infection generates ROS and activates Nrf2-mediated cytoprotective gene expression to improve cell survival. Furthermore, the report of Ivanov *et al*.^36^ claims transient expression of individual HCV proteins: core, E1, E2, NS4B and NS5A induces Nrf2 activation in a ROS-independent manner. The effect of core and NS5A-mediated Nrf2 activation was mediated by casein kinase 2 and PI3K pathway. A report by Carvajal-Yepes *et al*.^69^ claims that HCV infection inhibits Nrf2 gene transcription. This cytoprotective response seems important in the progression of HCC but the exact status of Nrf2 activation from acute to chronic HCV infection is unknown.

In this paper, we verified the role of ER-stress and UPR activation in a persistently HCV infected cell culture system using non-transformed and transformed hepatocytes. Our study shows that all three branches were nicely induced and the levels of UPR activation did not resolve over 18 to 20 days, suggesting that persistent HCV replication induces chronic ER-stress. We also found significant accumulation of reactive oxygen species (ROS) and oxidative stress in more than 90% of infected cells, which resulted in nuclear translocation of Nrf2 in 100% of infected cells starting from day 9 (22 days examined). The nuclear translocation of Nrf2 was prevented by PERK inhibitor or TUDCA, suggesting that PERK pathway activation is responsible for sustained nuclear translocation of Nrf2. Pretreatment of antioxidant α-tocopherol did not prevent nuclear translocation, suggesting that oxidative stress is not the main reason for nuclear translocation of Nrf2. We showed that silencing PERK pathway also inhibits Nrf2 activation in infected culture.

To understand the significance of Nrf2 activation on HCV related cancer mechanisms, we examined Nrf2-mediated induction of Mdm2 and degradation of Rb tumor suppressor. Silencing Nrf2 pathway also inhibited Mdm2 expression and restored Rb degradation. This stress induced Nrf2 activation and Mdm2-mediated Rb degradation was verified using Huh-7.5 cells treated with ER-stress inducer. Both PERK inhibitor and TUDCA decreased Nrf2 nuclear translocation, inhibited Mdm2 levels and restored Rb degradation. Silencing of Mdm2 by siRNA or inhibition of Mdm2 restored Rb degradation in HCV culture provides direct evidence of how ER-stress controls Rb and p53 degradation. Previous studies by Stanley Lemon’s group have shown that Rb degradation in HCV infected culture is mediated by direct binding of Rb with viral RNA-dependent RNA polymerase (NS5B)^70^. They also showed that NS5B-dependent ubiquitination of pRb and subsequent degradation via the proteasome and the degradation is mediated by ubiquitin ligase activity of E6-associated protein (E6AP)^71^. The loss of Rb function can also occur through the mutation in the Rb gene itself, hyper methylation of Rb promoter, bindings of viral proteins such as NS5B protein of HCV, E7 of the papilloma virus or E1A protein of adenovirus or post-transcriptional modification with tumor associated kinase activity^72^. Phosphorylation is also another well-characterized mechanism involved in Rb inhibition during cell cycle control, suggesting that Rb function can be inhibited by a wide variety of mechanisms^52^. In this study, we provide here another potential novel ER-stress related mechanism controlling Rb degradation through Mdm2 during HCV infection that leads to hepatocellular proliferation and chromosomal instability and HCC development **(**Fig. 11 **)**. Our results support the HCC mechanisms associated with alcoholic and non-alcoholic steatohepatitis (NASH), since these agents known to induce ER-stress during chronic liver disease. We show that the oncogenic Nrf2 nuclear translocation induced by ER-stress response associated with HCV is not inhibited by DAA-based antiviral treatment. Interferon-based antiviral therapy completely reverses the oncogenic Nrf2 nuclear translocation. These results indicate that interferon-based therapy provides additional cellular protection in addition to the antiviral clearance. IFN-mediated viral clearance reduces ER-stress and reverses the cellular distribution of Nrf2 suggesting the restoration of endogenous interferon levels after viral cure by DAA-based antiviral therapy is important to prevent HCC.

**Figure 11:** Hypothetical model illustrating the mechanism of oncogenic Nrf2 activation in chronic HCV infection due to ER-stress.
